The article "NAD(P)H: Quinone Oxidoreductase 1 Deficiency Conjoint with Marginal Vitamin C Deficiency Causes Cigarette Smoke Induced Myelodysplastic Syndromes" was retracted in 2026. Reasons: duplicated data; overlap with earlier publications; original data or images not available; unreliable results or conclusions.

# NAD(P)H: Quinone Oxidoreductase 1 Deficiency Conjoint with Marginal Vitamin C Deficiency Causes Cigarette Smoke Induced Myelodysplastic Syndromes

**DOI:** 10.1371/journal.pone.0020590

**Published:** 2011-05-31

**Authors:** Archita Das, Neekkan Dey, Arunava Ghosh, Tanusree Das, Indu B. Chatterjee

**Affiliations:** 1 Department of Biotechnology and Dr. B. C. Guha Centre for Genetic Engineering and Biotechnology, Calcutta University College of Science, Kolkata, West Bengal, India; 2 Infectious Diseases and Immunology Division, Indian Institute of Chemical Biology, Kolkata, West Bengal, India; Beth Israel Deaconess Medical Center, United States of America

## Abstract

**Background:**

The etiology of myelodysplastic syndromes (MDS) is largely unknown. Exposure to cigarette smoke (CS) is reported to be associated with MDS risk. There is inconsistent evidence that deficiency of NAD(P)H-quinone: oxidoreductase 1 (NQO1) increases the risk of MDS. Earlier we had shown that CS induces toxicity only in marginal vitamin C-deficient guinea pigs but not in vitamin C-sufficient ones. We therefore considered that NQO1 deficiency along with marginal vitamin C deficiency might produce MDS in CS-exposed guinea pigs.

**Methodology and Principal Findings:**

Here we show that CS exposure for 21 days produces MDS in guinea pigs having deficiency of NQO1 (fed 3 mg dicoumarol/day) conjoint with marginal vitamin C deficiency (fed 0.5 mg vitamin C/day). As evidenced by morphology, histology and cytogenetics, MDS produced in the guinea pigs falls in the category of refractory cytopenia with unilineage dysplasia (RCUD): refractory anemia; refractory thrombocytopenia that is associated with ring sideroblasts, micromegakaryocytes, myeloid hyperplasia and aneuploidy. MDS is accompanied by increased CD34(+) cells and oxidative stress as shown by the formation of protein carbonyls and 8-oxodeoxyguanosine. Apoptosis precedes MDS but disappears later with marked decrease in the p53 protein. MDS produced in the guinea pigs are irreversible. MDS and all the aforesaid pathophysiological events do not occur in vitamin C-sufficient guinea pigs. However, after the onset of MDS vitamin C becomes ineffective.

**Conclusions and Significance:**

CS exposure causes MDS in guinea pigs having deficiency of NQO1 conjoint with marginal vitamin C deficiency. The syndromes are not produced in singular deficiency of NQO1 or marginal vitamin C deficiency. Our results suggest that human smokers having NQO1 deficiency combined with marginal vitamin C deficiency are likely to be at high risk for developing MDS and that intake of a moderately large dose of vitamin C would prevent MDS.

## Introduction

Myelodysplastic syndromes (MDS) are a heterogeneous group of clonal hematological disease characterized by bone marrow hypercellularity, dysplasia, various degrees of cytopenia and a risk of progression to acute myeloid leukemia [1], [2]. MDS are divided into two groups, *de novo* and therapy related. Features of therapy related MDS include a myelodysplastic phase after the use of cytotoxic chemicals and/or radiotherapy for a malignant disease [2], [3]. *De novo* MDS is a disease of elderly people [4]. MDS patients have a poor survival. The genetic factor(s) and the environmental risk factor(s) leading to the increased susceptibility to MDS are poorly understood. Also one area that has not been explored is the influence of nutrition in MDS development [2].

The article "NAD(P)H: Quinone Oxidoreductase 1 Deficiency Conjoint with Marginal Vitamin C Deficiency Causes Cigarette Smoke Induced Myelodysplastic Syndromes" was retracted in 2026. Reasons: duplicated data; overlap with earlier publications; original data or images not available; unreliable results or conclusions.

Exposure to cigarette smoke (CS) and benzene are reported to be associated with MDS risk [5]–[10]. Risk from CS seems to be related to intensity and duration of smoking [2], [7], [11], [12]. In the case of benzene-induced MDS, the risk factor may be attributed to its metabolite p-benzoquinone (p-BQ), which targets to the bone marrow [5], [6]. Like that observed with benzene, the risk factor derived from CS for causing MDS may also be attributed to p-BQ. p-BQ is not present in CS, but it is apparently produced *in vivo* from p-benzosemiquinone (p-BSQ) of CS [13]–[15] by disproportionation [16] and oxidation by transition metal containing proteins [14]. p-BSQ is present in substantial amounts (100–200 µg/cigarette) in smoke from all commercial cigarettes examined as well as Kentucky research cigarettes [14], [17]. p-BQ is detoxified and thereby inactivated by NAD(P)H: quinone oxidoreductase 1 (NQO1), an enzyme ubiquitously present in all tissues, including the bone marrow [6], [18]–[20]. Normal NQO1 activity would protect individuals from p-BQ toxicity of the hematopoietic system. It is conceivable that NQO1 deficiency would increase one's risk of bone marrow toxicity. NQO1 deficiency is caused by polymorphism in NQO1^*^2, a single nucleotide change at position 609 of the NQO1 cDNA coding for a proline to serine change at position 187 in the amino acid structure of the protein [18]. A number of reports indicate that individuals with NQO1 deficiency may be at increased risk for the development of various forms of blood dyscrasia, including MDS and leukemia [6], [18], [21]–[23]. However, the results in different populations have not been consistent. A few reports show that lack of NQO1 activity does not correlate with increased risk of malignancy [24]–[26]. It is known that not all smokers have the risk for degenerative diseases. Only 15 per cent of the smokers are afflicted with diseases [27]. We considered that along with NQO1 deficiency, some other risk factor(s) might be involved in causing MDS.

The article "NAD(P)H: Quinone Oxidoreductase 1 Deficiency Conjoint with Marginal Vitamin C Deficiency Causes Cigarette Smoke Induced Myelodysplastic Syndromes" was retracted in 2026. Reasons: duplicated data; overlap with earlier publications; original data or images not available; unreliable results or conclusions.

Besides enzymatic detoxication by NQO1, p-BQ is strongly inactivated by vitamin C. Earlier we had reported that CS produces toxicity and tissue damage only in marginal vitamin C-deficient guinea pigs, but not in vitamin C-sufficient ones [14], [28]–[29]. We had previously indicated that a moderately large dose of vitamin C prevents CS-induced toxicity and tissue damage by reducing and thereby inactivating p-BQ [14]. We therefore considered that in addition to NQO1 deficiency, the nutritional status of vitamin C might be a critical determining factor for causing CS-induced MDS.

Understanding the relationship among CS exposure, NQO1 deficiency and marginal vitamin C deficiency in population-based studies is problematic. We have addressed this relationship using a guinea pig model. Here we show that CS exposure produces MDS only when the guinea pigs have deficiency of NQO1 conjoint with marginal vitamin C deficiency. MDS are not produced in singular deficiency of either NQO1 or marginal vitamin C deficiency. Also, MDS do not occur in vitamin C-sufficient guinea pigs.

## Results

### Vitamin C status in plasma and bone marrow

We have produced marginal vitamin C deficiency in guinea pigs (350–450 g body weight) by feeding them 0.5 mg vitamin C/day. Vitamin C sufficient guinea pigs were fed 15 mg vitamin C/day. The minimum dose of vitamin C needed to maintain the guinea pigs without onset of scurvy is 0.15 mg/100 g body weight [30]. At the dosage of 0.5 mg/day/350–450 g body weight, no scurvy symptom appeared up to a period of 8 weeks. Table 1 shows that after feeding vitamin C-deficient diet at a dose of 0.5 mg/day for 21days, the vitamin C levels are very low in the plasma and bone marrow of guinea pigs that are not detectable after exposure to CS. This is apparently because CS consumes vitamin C [29]. When the guinea pigs were fed 15 mg vitamin C/day, the vitamin C contents of plasma and bone marrow were adequate.

**Table 1:** Vitamin C levels in the plasma and bone marrow of guinea pigs fed 0.5 mg/day and 15 mg/day vitamin C for 21 days and exposed to air or CS.

	Vitamin C level			
	Plasma (mg/100 ml)		Bone marrow (µg/10^8^ cells)	
	Vitamin C supplementation/day			
Group	0.5 mg	15 mg	0.5 mg	15 mg
**Air**	0.12±0.01*	0.67±0.04	0.18±0.02	5.17±0.29
**DC**	0.14±0.01	0.89±0.02	0.13±0.01	2.27±0.06
**CS**	ND	0.44±0.12	ND	2.65±0.20
**DC+CS**	ND	1.27±0.20	ND	2.75±0.10

Dietary supplementation of vitamin C 0.5/15 mg/day) was initiated after deprivation of the vitamin for 7 days. The vitamin C contents of plasma and bone marrow were estimated on day 21^st^ by HPLC as described under Materials and Methods. ND means not detectable. * Data represent mean ±S.D. (n = 4).

The article "NAD(P)H: Quinone Oxidoreductase 1 Deficiency Conjoint with Marginal Vitamin C Deficiency Causes Cigarette Smoke Induced Myelodysplastic Syndromes" was retracted in 2026. Reasons: duplicated data; overlap with earlier publications; original data or images not available; unreliable results or conclusions.

### Bone marrow NQO1 activity

NQO1 deficiency was produced by feeding an aqueous suspension of dicoumarol [3,3′-methylene-bis(4-hydroxycoumarine), Sigma, USA], an inhibitor of NQO1 [31]. Figure 1A shows that feeding dicoumarol (DC) at a dose of 3 mg/day for 21 days produces about 90% inhibition of NQO1 activity in the bone marrow of guinea pigs. The decrease in the NQO1 activity took place gradually up to 21 days of the experimental period (Figure 1B). Western blot analysis shows that there is no significant change in the NQO1 gene expression at the protein level (Figure S1).

**Figure 1:** NQO1 Activity of bone marrow cells of guinea pigs fed 0.5 mg or 15 mg vit C/day. (Panel A) AIR, exposed to air; DC, fed 3 mg DC/day; CS, exposed to CS; DC+CS, fed 3 mg DC/day and exposed to CS. * indicates significant difference (p<0.05) with respect to air exposed guinea pigs.(Panel B) NQO1 activity at different time periods of DC+CS group. * indicates significant difference (p<0.05) with respect to 0 day. Bars over the respective columns represent means ± SD (n = 6), Vit C means vitamin C.

### Occurrence of MDS in guinea pigs as evidenced by morphology, histology and cytogenetic studies

One important method of diagnosis of MDS relies on morphologic assessments based on World Health Organization (WHO) classification [32]. Here we have diagnosed MDS in guinea pigs on the basis of bone marrow cell morphology, histology and cytogenetic examinations. The guinea pigs were divided into 8 groups (6 animals/group): (i) 0.5 mg vitamin C and exposed to air (sham controls), (ii) 0.5 mg vitamin C and exposed to CS, (iii) 0.5 mg vitamin C fed DC and exposed to air, (iv) 0.5 mg vitamin C fed DC and exposed to CS, (v) 15 mg vitamin C and exposed to air, (vi) 15 mg vitamin C and exposed to CS, (vii) 15 mg vitamin C fed DC and exposed to air, and (viii) 15 mg vitamin C fed DC and exposed to CS. All the guinea pigs of groups (i–iii) and (v–viii) were fed with respect to the average food consumption of the guinea pigs of group (iv). After exposure to CS for 21 days, MDS were produced only in the guinea pigs having deficiency of NQO1 conjoint with marginal vitamin C deficiency. Figure 2A, V and IX show that in comparison to normal segmented neutrophils (Figure 2AI), there are hyper segmented neutrophils (7 lobes) in the blood film of MDS guinea pigs. These observations indicate dysgranulopoiesis, as reported by others [33]. Figure 2AXIII depicts poorly functioning large platelets in the MDS guinea pigs, as compared to the platelets observed in the blood film of guinea pigs fed 0.5 mg vitamin C/day and exposed to air (Figure 2AI). In contrast to all other experimental groups there was significant decrease in the number of platelets in the MDS guinea pigs (Table S1). All these various changes were observed in the MDS guinea pigs, but not in any of the guinea pigs other than MDS, including vitamin C-sufficient guinea pigs fed 15 mg vitamin C/day (Figure 2A XVII).

The article "NAD(P)H: Quinone Oxidoreductase 1 Deficiency Conjoint with Marginal Vitamin C Deficiency Causes Cigarette Smoke Induced Myelodysplastic Syndromes" was retracted in 2026. Reasons: duplicated data; overlap with earlier publications; original data or images not available; unreliable results or conclusions.

**Figure 2:** Identification of MDS in guinea pigs by blood and bone marrow cell morphology, measurement of CD34(+) cells and cytogenetic studies. (Panel **A**) Differential staining showing some typical changes in blood and bone marrow cell morphology of MDS guinea pigs and its prevention by feeding the animals 15 mg vitamin C/day. **A, I–IV**, represent sham controls (fed 0.5 mg vitamin C/day and exposed to air); **A, V–XVI**, represent MDS guinea pigs (CS-exposed fed DC and 0.5 mg vitamin C/day); **A, XVII–XX**, represent CS-exposed guinea pigs fed DC and 15 mg vitamin C/day. Blood smear - Leishman stain; bone marrow aspirate - Wright Geimsa stain, except Perls' stain in X and XIV; (magnification 400×, except I, V, VI, IX, XIII, XVII; 1000× magnification). → indicates dysplastic cells. Vit C means vitamin C. (Panel B) Measurement of CD34(+) cells in bone marrow by flow cytometry. (Panel **C**) Quantitative evaluation of CD34(+) cells; bars (means ± SD, n = 6) over the respective columns represent CD34(+) cells, * significantly different (p<0.05) with respect to 1–7 samples. (Panel D) Geimsa-stained metaphase spread showing aneuploidy in **II**; (magnification 1000×).

MDS are usually present with myeloid hyperplasia in the bone marrow [34]. However, some types have erythroid predominance such as RA and RARS (32). We also observed that the myeloid to nonmyeloid ratio increased 4 fold (p<0.05) in the bone marrow of MDS guinea pigs compared to the guinea pigs of all others groups. The ratio increased gradually up to 21 days of the experimental period (Table S2 and Figure S2A). However the guinea pigs exposed to cigarette smoke only without the addition of vitamin C show no myeloid hyperplasia (Table S2 and Figure S2A). There was no change in the WBC count in the blood, but RBC and hemoglobin were significantly decreased (p<0.05, n = 6) in the MDS guinea pigs (Table S1). Morphologically, dysplasia was seen in all the lineages with predominance in the erythroid and granuloid lineages. Quantitation of dysplasia indicate: dysplasia in 15% of the cells in the erythroid lineages, 9.5% in the granuloid lineage and 8% in the megakaryocytic lineage. Figure 2AII shows normal megaloblast, a large cell with dark blue cytoplasm and primitive nuclear chromatin pattern in guinea pigs fed 0.5 mg vitamin C/day and exposed to air. In contrast to this, Figure 2AVI depicts marked hyper- cellular vacuolation with some megaloblastoid changes and Figure 2AX shows ring sideroblasts. Many blue siderotic granules were surrounding the nucleus, as evidence of dyserythropoiesis found in MDS guinea pigs [33]. It has been reported that pathologic iron accumulation occurs in the erythroblasts as evidence of dyserythropoiesis in MDS [35], [36]. Figure 2AXIV depicts blue spots (Perls' stain) in the bone marrow of MDS guinea pigs that represent iron accumulation as evidence of dyserythropoiesis. The dyserythropoiesis was prevented in CS-exposed NQO1-deficient guinea pigs by feeding the animals 15 mg vitamin C/day (Figure 2AXVIII).

The article "NAD(P)H: Quinone Oxidoreductase 1 Deficiency Conjoint with Marginal Vitamin C Deficiency Causes Cigarette Smoke Induced Myelodysplastic Syndromes" was retracted in 2026. Reasons: duplicated data; overlap with earlier publications; original data or images not available; unreliable results or conclusions.

In granuloid lineage, Figure 2AIII depicts normal neutrophilic myelocyte with eccentric nucleus and faint cytoplasm. Compared to this, bone marrow of MDS guinea pig shows dysplastic myelocyte indicating abnormal separation of nuclear lobes (Figure 2AVII) and atypical mononuclear cells with altered nuclear and cytoplasm ratio (Figure 2AXI). This suggests dysgranulopoiesis in MDS. Dysgranulopoiesis did not occur in guinea pigs fed 15 mg vitamin C/day (Figure 2AXIX). Figure 2AXV depicts myeloblast, the first recognizable cell of the granuloid series. The percent of myeloblast increased considerably in the MDS guinea pigs. In the guinea pigs fed 0.5 mg vitamin C and exposed to air, the myeloblast count has been found to be 1.98%±0.43 (p<0.05, n = 6), whereas that in the MDS guinea pigs is 4.88%±0.63 (p<0.05, n = 6). Bone marrow hematopoietic progenitor cells are a heterogeneous population with varying degree of maturation in several cell lineages. It is reported that CD 34(+) cell population is increased in MDS [36], [37]. Using flow cytometry analyses, here we show that the percentage of CD 34(+) cells in the bone marrow of MDS guinea pigs has increased significantly (p<0.05, n = 6) about 10% over that observed in the bone marrow of guinea pigs fed 0.5 mg of vitamin C and exposed to air. No increase in the CD 34(+) cells was observed in other experimental groups (Figure 2B and C).

Also, compared to the all others groups the number of megakaryocytes increased significantly (p<0.05, n = 6) in the MDS guinea pigs. However, the platelet count decreased (p<0.05, n = 6) (Table S1). This indicates occurrence of micromegakaryocytes (Figure 2A, VIII, XII), which are seen in MDS animal and sterile dysplastic megakaryocytes (Figure 2A XVI) that evidences dysmegakaryopoiesis as reported by others [33]. Figure 2A, IV and XX show normal megakaryocytes.

Previous study had demonstrated that hypercellularity in the bone marrow is a characteristic feature of MDS [38]. Using hematoxylin and eosin (H&E) staining here we show that compared to that observed in guinea pigs of other experimental groups, including those fed 15 mg vitamin C/day, there is significant (p<0.05, n = 6) increase of bone marrow cellularity in the MDS guinea pigs (Figure S2B II). However, there was no increase in bone marrow cellularity in the guinea pigs exposed to cigarette smoke only without addition of vitamin C (Figure S2B IV). The quantitation of cellularity was made by numerical counting using Dewinter Biowizard 4.1 software.

The article "NAD(P)H: Quinone Oxidoreductase 1 Deficiency Conjoint with Marginal Vitamin C Deficiency Causes Cigarette Smoke Induced Myelodysplastic Syndromes" was retracted in 2026. Reasons: duplicated data; overlap with earlier publications; original data or images not available; unreliable results or conclusions.

Numerical chromosomal aberrations, aneuploidy, are common in cancer including hematopoietic tumor cells [39]. We have observed aneuploidy in the MDS guinea pigs (Figure 2CII). The number of chromosomes in normal guinea pigs is 62, karyotype 60+XY [40]. In MDS guinea pigs, the number varied from 116 to 128. A critical analyses of 100 metaphases revealed that 70% metaphases represented normal karyotype, whereas 30% metaphases represented aberrations in MDS guinea pigs. No such aberration occurred in CS-exposed NQO1–deficient guinea pigs fed 15 mg vitamin C/day (Figure 2CIII).

All the aforesaid results indicate that the MDS occur only in CS-exposed guinea pigs having deficiency of NQO1 conjoint with marginal vitamin C deficiency. Such pathophysiological events did not occur in any of the experimental groups other than MDS. Nevertheless, as mentioned before supplementation of a moderately high dose of vitamin C (15 mg/day) prevented the myelodysplastic changes in CS-exposed NQO1-deficient guinea pigs.

The aforesaid results have been presented using Kentucky research cigarettes 3R4F. In separate experiments, using a commercial cigarette (Wills Navy Cut, ITC, India), similar MDS was diagnosed on the basis of morphology, histology and cytogenetics (data not shown). This was done to show that Kentucky research cigarette was not specific.

### Apoptosis in the guinea pig bone marrow cells

It is reported that apoptosis is an early event in MDS and ineffective hemaptopoiesis found in MDS is caused by an increased incidence of apoptosis in bone marrow cells [41]. Here we show that MDS is preceded by apoptosis of the bone marrow cells. Apoptosis has been evidenced by TUNEL assay, flow cytometry analysis using Annexin V/PI staining, phosphorylation of p53, activation of caspase 3 and increase in the bax/Bcl-2 ratio as well as up regulation of TNF-α and cleavage of caspase 8.

Figure 3, A and B show that in the guinea pigs fed 0.5 mg vitamin C and 3 mg DC/day, there is progressive increase in the number of TUNEL positive cells in the bone marrow after exposure to CS for 7 and 14 days. However, after continuation of CS exposure for 21 days, the TUNEL positive cells have disappeared, which is accompanied by occurrence of MDS. The TUNEL positive cells are also absent when the DC-treated CS-exposed guinea pigs are fed 15 mg vitamin C/day. Since 15 mg vitamin C prevents MDS (Figure 2), the results would indicate that a moderately high dose of vitamin C prevents apoptosis and MDS.

The article "NAD(P)H: Quinone Oxidoreductase 1 Deficiency Conjoint with Marginal Vitamin C Deficiency Causes Cigarette Smoke Induced Myelodysplastic Syndromes" was retracted in 2026. Reasons: duplicated data; overlap with earlier publications; original data or images not available; unreliable results or conclusions.

**Figure 3:** Assessment of apoptosis by TUNEL assay, flow cytometry and cell signaling in bone marrow cells of guinea pigs. (Panel A) TUNEL assay of bone marrow cells. The rows were stained with fluorescein labeled dUTP and 4, 6-diamidino-2-phenylindole (DAPI), respectively; green fluorescence indicates TUNEL positive cells (magnification 200×). (Panel B) Quantitative evaluation of TUNEL positive cells; bars (means ± SD, n = 6) over the respective columns represent TUNEL positive cells, * significantly different (p<0.05) with respect to 0 day, ** significantly different (p<0.05) from 14 days treatment. (Panel **C**) Flow cytometry analyses of bone marrow cells using Annexin V-FITC fluorescence (Y-axis) vs PI (X-axis); quadrants: lower left, viable cells; upper left, apoptotic cells; upper right, late apoptotic and lower right, necrotic cells. (Panel D) p53 status in the bone marrow cells at different time. (Panel E) and (Panel F) Immunoblots of p-p53 (phospho-p53), Bax, Bcl-2, caspase 3 (C3), cleaved caspase 3 (CC3). (Panel G) and (Panel H) Immunoblots of TNF-α, caspase 8 (C8) and cleaved caspase 8 (CC8). Vit C means vitamin C.

As observed by TUNEL assay, flow cytometry analysis shows (Figure 3C) that in the DC-treated CS-exposed guinea pigs fed 0.5 mg vitamin C, the apoptotic population (Annexin V +/PI −) is maximum (24.52%) on day 14 and absent on day 21 (0.12%). The percentage of necrosis is negligible.

That MDS is preceded by apoptosis is also evidenced by an increase in the p53 level in the bone marrow cells on day 14 (Figure 3D, row 4), which is accompanied by an increase in phosphorylated p53 (Figure 3F, row 1). After exposure to CS, the p53 levels were comparatively higher on days 14 and 21 than those observed on days 0 and 7 (Figure 3D, row 3). However, after treatment with DC along with CS, the p53 levels were high on days 7 and 14 but very low on day 21 (Figure 3D, row 4), when apoptosis was absent and MDS appeared. This is supported by the observation that while p-p53 level was high on day 14 when apoptosis was high, it was absent on day 21 (Figure 3F, row 1) when apoptosis disappeared and MDS appeared. Apoptosis is further supported by an increase in the levels of Bax (not Bcl-2), caspase 3, cleaved caspase 3 on day 14 that decreased in the MDS guinea pigs on day 21 (Figure 3F, rows 2, 3, 4 and 5, respectively).

The article "NAD(P)H: Quinone Oxidoreductase 1 Deficiency Conjoint with Marginal Vitamin C Deficiency Causes Cigarette Smoke Induced Myelodysplastic Syndromes" was retracted in 2026. Reasons: duplicated data; overlap with earlier publications; original data or images not available; unreliable results or conclusions.

It had been reported that in early MDS increased apoptosis is partially due to up regulation of TNF-α and death receptors [36]. Here we show that the levels of TNF-α and its downstream effector cleaved caspase 8 are markedly increased on day 14. TNF-α decreased considerably and cleaved caspase 8 was practically absent in the MDS guinea pigs on day 21 (Figure 3H, rows 1 and 3, respectively). Apoptosis was absent in all the experimental groups other than MDS as well as in the guinea pigs fed 15 mg vitamin C/day (Figure 3E and G).

Activation of epidermal growth factor receptor (EGFR) has been implicated in the pathogenesis of a variety of malignancies including leukemia. Reports also indicate that the Akt pathway is critical for cell survival and proliferation in high-risk MDS patients. We have also observed activation of EGFR, MAPK/Ras pathway as well as Akt in MDS produced in the guinea pigs (Figure S3).

### p-BQ-protein adduct and oxidative stress in MDS

CS contains substantial amount of p-BSQ, [15], [17] a major long-lived radical. We had shown before that p-BSQ is oxidized to p-BQ by transition metal containing proteins [14]. The amount of p-BQ calculated to be formed in the lungs from the inhaled cigarette smoke is 22.5 µg/day (Supporting Information Text S1). Using antibody against p-BQ and immunoblotting, here we show that bone marrow proteins of marginal vitamin C-deficient CS-exposed guinea pigs contain p-BQ-protein adducts (Figure 4, A and B). Also, incubation of bone marrow cells *in vitro* with p-BQ or aqueous extract of cigarette smoke (AECS) produced p-BQ-protein adducts (Figure 4C). This would indicate that probably one mechanism of CS-induced MDS is p-BQ-induced modification of bone marrow proteins. The formation of p-BQ-protein adduct is prevented by vitamin C (15 mg/day) (Figure 4A). p-BQ is also a redox cycling agent [42]. The reactive oxygen species (ROS) generated by redox cycling lead to the formation of protein carbonyls as well as 8-oxo-7, 8-dihydroguanosine (8-oxodG) that are associated with carcinogenesis [42]. As depicted in Figure 4D, bone marrow cells of DC-treated vitamin C-deficient guinea pig show increase in ROS at day 14 of CS-exposure, which is decreased after continuation of exposure for 21 days. The oxidative stress is further demonstrated by measuring protein carbonyl, an evidence of protein oxidation, (Figure 4E) and 8-oxodG, an evidence of DNA oxidation (Figure 4, F and G). No ROS was produced in the guinea pigs fed 15 mg vitamin C (Figure 4D), indicating that moderately high dose of vitamin C prevents CS-induced oxidative stress.

**Figure 4:** Identification of p-BQ-protein adducts and detection of oxidative stress in bone marrow cells of guinea pigs. (Panel A) p-BQ protein adducts in the bone marrow cells of CS-exposed guinea pigs on day 21 *in vivo*. (Panel B) p-BQ protein adducts in CS-exposed guinea pigs at different time period *in vivo*. (Panel **C**) p-BQ protein adducts formed in marrow cells *in vitro* after incubation with p-BQ and AECS (aqueous extract of cigarette smoke), respectively; M, marker (cropped). (Panel D) ROS production in MDS guinea pigs at different time periods, as evidenced by flow cytometry. The X-axis represents the intensity of dichlorodihydrofluorescein diacetate (H_2_DCFDA). (Panel E) Protein oxidation as evidenced by oxyblot indicating formation of protein carbonyl. (Panel F) DNA oxidation as evidenced by the formation of 8-oxodG; upper row: green fluorescence indicates formation of 8-oxodG; lower row: stained with DAPI; (magnification 200×). (Panel G) Quantitative evaluation of 8-oxodG; * indicates significant difference from 0 and 7 days. Vit C means vitamin C.

The article "NAD(P)H: Quinone Oxidoreductase 1 Deficiency Conjoint with Marginal Vitamin C Deficiency Causes Cigarette Smoke Induced Myelodysplastic Syndromes" was retracted in 2026. Reasons: duplicated data; overlap with earlier publications; original data or images not available; unreliable results or conclusions.

### MDS produced in the guinea pigs are irreversible

It is known that MDS is an irreversible condition caused in some cases by genotoxicity. Here we show that MDS produced in the guinea pigs are irreversible, as evidenced by bone marrow cell morphology and cytogenetic examination. Six guinea piga were fed 0.5 mg vitamin C and 3 mg DC/animal/day and exposed to CS. Another 6 guinea pigs were fed 0.5 mg vitamin C/animal/day and exposed to air (sham controls). After exposure to CS for 21 days, 2 out of the 6 guinea pigs were sacrificed and MDS diagnosed by morphology and cytogenetic examination described before in the text. CS exposure was discontinued in the remaining 4 guinea pigs and they were fed 15 mg vitamin C/animal/day. Supplementation of DC (3 mg/day) was continued for maintaining NQO1 deficiency. After 6 days, there was drastic fall in the food intake and loss of body weight. At that stage, the animals were sacrificed and blood smear, bone marrow cell morphology, CD34(+) cell count and cytogenetic examination were performed. We have also measured NQO1 activity and the p53 status in the bone marrow. Figure 5A a, b, c, d show normal morphology in blood and bone marrow cells. In contrast to these, Figure 5A e and f depict poor functioning large platelets and dyserythropoietic changes in bone marrow cells. Figure 5A g and h show micromegakaryocyte and ring sideroblast. The percentage of CD34(+) cells in the bone marrow increased significantly (p<0.05, n = 4) about 22% over that observed in the sham controls (Figure 5B). Here we have also observed anuploidy, the number varied from 104 to 120 (Figure 5C). A critical analyses of 100 metaphases revealed that 62% metaphases represented normal karyotype, (Figure 5C) whereas 38% metaphases represented anuploidy (Figure 5C). All these aforesaid results indicate that the animals had persistent changes confirming irreversibility of MDS produced in the guinea pigs. Figure 5D shows 90% inhibition of NQO1 activity in the bone marrow without any change in the NQO1 gene expression at the protein level (Figure 5E, row 1). However, the p53 level was markedly low in the MDS guinea pigs fed 15 mg vit C (Figure 5E, row 2).

The article "NAD(P)H: Quinone Oxidoreductase 1 Deficiency Conjoint with Marginal Vitamin C Deficiency Causes Cigarette Smoke Induced Myelodysplastic Syndromes" was retracted in 2026. Reasons: duplicated data; overlap with earlier publications; original data or images not available; unreliable results or conclusions.

**Figure 5:** MDS produced in the guinea pigs are irreversible. (Panel **A**) Differential staining showing persistent changes in blood and bone marrow cell morphology of MDS guinea pigs followed by discontinuation of CS exposure and feeding 15 mg vitamin C/day. **A, a–d**, represent sham controls (fed 0.5 mg vitamin C/day and exposed to air); **A, e–h**, represent MDS guinea pigs followed by discontinuation of CS exposure and feeding 15 mg vitamin C/day. Blood smear - Leishman stain; bone marrow aspirate - Wright Geimsa stain, except Perls' stain in **d and h**; (magnification 400×). (Panel **B**) Measurement of CD34(+) cells in bone marrow by flow cytometry. (Panel **C**) Geimsa-stained metaphase spread showing aneuploidy in MDS guinea pigs followed by discontinuation of CS exposure and feeding 15 mg vitamin C/day; (magnification 1000×). (Panel **D**) NQO1 Activity of bone marrow cells. Bars over the respective columns represent means ± SD (n = 4); * indicates significant difference (p<0.05, n = 4) with respect to air exposed guinea pigs. (Panel **E**) NQO1 and p53 status in the bone marrow cells.

## Discussion

MDS represents a malignant entity that shares many characteristics with acute myeloid leukemia (AML). Approximately one-third of patients ultimately progress to AML [43]. MDS is 3–4 times more prevalent than AML and follows a more indolent course [43]. The etiology of MDS is yet to be known in most patients. However, intrinsic defects in hematopoietic cells and extrinsic factors affecting bone marrow microenvironment are involved in the pathogenesis of this disorder. One such extrinsic factor is cigarette smoke. In this paper we have shown that CS exposure mimics MDS in guinea pigs having deficiency of NQO1 conjoint with marginal vitamin C deficiency. Singular deficiency of NQO1 or marginal vitamin C deficiency does not produce CS-induced MDS. We have used the guinea pig as a model animal because, like human, it is incapable of synthesizing vitamin C and is dependent on the dietary source of the vitamin [44], [45]. Also, the guinea pig has anatomical and CS-induced pathophysiological similarities to humans [46].

The article "NAD(P)H: Quinone Oxidoreductase 1 Deficiency Conjoint with Marginal Vitamin C Deficiency Causes Cigarette Smoke Induced Myelodysplastic Syndromes" was retracted in 2026. Reasons: duplicated data; overlap with earlier publications; original data or images not available; unreliable results or conclusions.

According to the WHO classification, [32] the MDS produced in the guinea pigs fall in the category of refractory cytopenia with unilineage dysplasia (RCUD): refractory anemia (RA); refractory thrombocytopenia (RT). This has been evidenced by blood findings of bicytopenia but no blast. Bone marrow findings indicate unilineage dysplasia in >10% of the cells in one myeloid lineages (15% erythroid, 9.5% granuloid, 8% megakaryocytic lineages) and <5% blasts (4.88%±0.63 SD). Also, less than 15% erythroid precursors are ring sideroblasts (6.0%). Perls' stain showed blue spots in marrow cells indicating iron accumulation. MDS is also accompanied by micromegakaryocyte. Because three lineages are affected, the disorders probably occurred at the pluripotent stem cells. The abnormalities in hematopoiesis are accompanied by an increase in hematopoietic precursor cells (CD34+). We have also observed anueploidy in MDS guinea pigs, indicating genomic instability. The MDS produced in the guinea pigs are irreversible as evidenced by bone marrow cell morphology, CD34 (+) cell count and cytogenetic studies.

Until now the risk factor(s) in CS responsible for producing MDS has remained unclear. CS contains about 4000 compounds [47], including a number of carcinogens [48] and semiquinones [14], [15]. Among the carcinogens, the most extensively studied compounds are benzo[a] pyrene (BP) and 4-(methylnitrosamino)-1-(3-pyridil)-1-butanone (NNK) [49]. The concentrations of these in smoke from one cigarette are very low: 20–40 ng (BP) and 80–960 ng (NNK), respectively [48], [49]. Moreover, the carcinogenic effects of both these compounds are organospecific. They produce only lung tumor at very high doses [48]. We consider that the apparent risk factor derived from CS for producing MDS is p-BQ. CS does not contain p-BQ. p-BQ is produced from p-BSQ, which is present in CS in substantial amounts depending on the brand of the cigarette (100–200 µg/cigarette) [14], [15], [17]. p-BSQ is converted to p-BQ by disproportionation: 2p-BQ→p-BQ+Hydroquinone [16] as well as oxidation by transition metal (M) containing proteins: p-BSQ+M^ox^−Protein→p-BQ+M^red^−Protein [14]. p-BQ derived from p-BSQ of CS gets into the bloodstream and goes to the bone marrow, the target organ [5], [6], where it interacts with ε-amino groups of lysine residues of proteins forming covalent adducts [14], [50]. Using antibody to p-BQ and western blot, here we have demonstrated formation of p-BQ-protein adducts in the bone marrow cells of CS-exposed guinea pigs. However, how p-BQ causes MDS is not clear. It has been proposed for benzene-induced leukemia that p-BQ derived from benzene causes damage to tubulin, histone proteins, topoisomerase II leading to DNA strand break, mitotic recombination and aneuploidy in stem cells or early progenitor cells leading to leukemia [5].

p-BQ is also a redox cycling agent [42] that generates ROS leading to the formation of protein carbonyl as well as 8-oxodG. Elevated levels of 8-oxodG were found in a significant proportion of MDS patients, indicating increased oxidative DNA damage or defective handling of oxidative load [51]. In recent years the biomarker 8-oxodG has become pivotal for measuring the effect of endogenous oxidative damage to DNA and as a factor influencing the initiation and promotion of carcinogenesis [52], [53]. 8-oxodG is a potent mutagen. Once incorporated into DNA, it codes for error prone DNA synthesis [54]. We have documented the formation of ROS, protein carbonyl as well as 8-oxodG in the bone marrow cells of MDS guinea pigs.

The article "NAD(P)H: Quinone Oxidoreductase 1 Deficiency Conjoint with Marginal Vitamin C Deficiency Causes Cigarette Smoke Induced Myelodysplastic Syndromes" was retracted in 2026. Reasons: duplicated data; overlap with earlier publications; original data or images not available; unreliable results or conclusions.

We have shown that CS-induced MDS is produced only when the guinea pigs have NQO1 deficiency conjoint with marginal vitamin C deficiency. The function of vitamin C (E′° = +0.08 V) is to reduce p-BQ (E′° = +0.71V) to the less toxic HQ, which is excreted as sulfate and glucuronide. Although a function of NQO1 is also to reduce p-BQ, [6], [18]–[20] we consider that NQO1 has some other function than only to reduce and inactivate p-BQ. One prominent function of NQO1 is to regulate the stability of p53. NQO1 binds with p53 and stabilizes it [55]. We have produced NQO1 deficiency in the guinea pigs by feeding them DC, a potent inhibitor of NQO1 [55], [56] The crystal structure of human NQO1 in complex with DC determined at 2.75 Å resolution shows that DC competes with NAD(P)H for binding to NQO1 and thereby inhibits NQO1 activity [57]. The NQO1-dicoumarol complex disrupts NQO1-p53 binding and induces ubiquitin-independent proteasomal degradation of p53 [58]. However, here we show that although there is some decrease in the p53 protein after treatment with DC (Figure 3D, row 2), there is a marked decrease of p53 after treatment with DC along with CS. (Figure 3D, row 4). The possibility that p-BQ derived from CS formed adduct with p53 resulting in proteolytic degradation of the protein [14] is eliminated, because there is no loss of p53 after CS treatment (Figure 3D, row 3). The mechanism of marked decrease of p53 accompanied by disappearance of apoptosis and appearance of MDS is not clear at present. p53 is a tumor suppressor protein that can induce apoptosis and cell cycle arrest and thereby prevent accumulation of DNA-damaged cells that could lead to the development of cancer [31], [59]. We consider that loss of p53 may be associated with the development of MDS. Cells lacking p53 are at high risk for malignant transformation and easily become aneuploid [59]. So, one of the causes of aneuploidy observed in MDS guinea pigs may be decrease in the p53 protein level.

The article "NAD(P)H: Quinone Oxidoreductase 1 Deficiency Conjoint with Marginal Vitamin C Deficiency Causes Cigarette Smoke Induced Myelodysplastic Syndromes" was retracted in 2026. Reasons: duplicated data; overlap with earlier publications; original data or images not available; unreliable results or conclusions.

Vitamin C has a long and controversial history in the prevention and treatment of cancer. In an experiment on guinea pigs, it was shown that methylcholanthrene induced tumors sooner in the animals deficient in vitamin C as compared to those fed adequate amount of vitamin C [60]. Several epidemiological studies have pointed to the importance of dietary and Supporting vitamin C in the prevention of various types of cancer, including leukemia [61], [62]. In leukemic patients, the plasma levels of vitamin C were practically undetectable [63]. A number of recent papers show that pharmacological doses of vitamin C decreases growth and weight of human, rat and murine tumor xenografts in athmyc, nude mice [64]. Results indicate that high doses of vitamin C are safe and well tolerated in different patients [64].

We have observed that MDS is preceded by apoptosis of marrow cells. Apoptosis is a well recognized phenomenon in early MDS [36], [38], [65], [66]. It is reported that caspase 3 activity is especially enhanced in early MDS and declined in late MDS and absent in leukemia [66]. In MDS guinea pigs, we have observed both intrinsic pathways of apoptosis involving Bax, Bcl-2 and caspase 3 as well as extrinsic pathway involving TNF-α and caspase 8. A higher expression of TNF-α has actually been found in MDS that correlates with apoptosis [36]. Marked apoptosis is observed on day 14 in the bone marrow cells of CS-exposed guinea pigs having deficiency in NQO1 and marginal vitamin C deficiency. Apoptosis disappears on day 21, which is accompanied by occurrence of MDS. Apparently the cells that escape apoptosis survive and proliferate to produce hypercellularity and MDS. In the MDS guinea pigs, increased cellular proliferation has probably occurred via activation of EGFR, Ras/MAPK pathway as well as Akt (Supporting Results in Text S1). It is reported that CS-induced persistent activation of EGFR, ERK1/2 and Akt results in cell proliferation and transformation [67].

In conclusion, our results suggest that three factors combined together lead to CS-induced MDS: exposure to CS, NQO1 deficiency and marginal vitamin C deficiency. MDS is not produced in vitamin C-sufficient guinea pigs fed a moderately high dose of vitamin C. However, after the onset of MDS vitamin C becomes ineffective. Like that observed in humans, MDS produced in the guinea pigs are irreversible. If the results obtained with guinea pigs are applicable to human, smokers having NQO1 deficiency conjoint with marginal vitamin C deficiency would be at high risk for developing MDS. Nevertheless, intake of a moderately high dose of vitamin C should prevent occurrence of MDS in smokers.

The article "NAD(P)H: Quinone Oxidoreductase 1 Deficiency Conjoint with Marginal Vitamin C Deficiency Causes Cigarette Smoke Induced Myelodysplastic Syndromes" was retracted in 2026. Reasons: duplicated data; overlap with earlier publications; original data or images not available; unreliable results or conclusions.

## Materials and Methods

### Animals

Male short hair guinea pigs weighing 350–450 g were divided into weight-matched groups and fed vitamin C-free diet (Supporting Information Text S1) for one week to minimize the vitamin C level of tissues [28]. After 1 week, the guinea pigs were fed either vitamin C-deficient (0.5 mg/day) or vitamin C-sufficient diet (15 mg/day) [29].

### Ethics Statement

All methods were approved by the Institutional Animal Ethics Committee, Permit No. 797/CPCSEA, Department of Biochemistry, University of Calcutta. All efforts were made to minimize suffering of the animals.

### Exposure to cigarette smoke

The guinea pigs were subjected to cigarette smoke exposure from 5 Kentucky Research cigarettes 3R4F (2 puffs per cigarette)/animal/day (6 days/week) in a smoke chamber, as described before [14], except that the time of exposure was 90 seconds instead of 45 seconds (for details, see Supporting Information Text S1). Pair-fed sham controls were subjected to air exposure instead of CS under similar conditions. After the experimental period, the animals were euthanized under deep anesthesia using i.p. injection of ketamine hydrochloride (100 mg/kg body weight) and thereafter the respective tissues were excised.

### Measurement of vitamin C

Vitamin C was measured by HPLC as described before [14], except that 0.13 mM ß-mercaptoethanol was added to the plasma and bone marrow lysate to prevent oxidation of vitamin C.

### Bone marrow NQO1 activity and protein

Bone marrow was homogenized in a buffer containing 50 mM Tris-HCl ph7.4, 250 mMsucrose, 1 mM EDTA [21] and cytosol prepared by centrifuging at 19000 g for 15 minutes. The cytosolic fraction (75 µg protein) was analyzed for NQO1 activity following the decrease in NADH absorbance at 340 nm in a UV-2450 UV-VIS spectrophotometer (Shimadzu) [31]. NQO1 protein was measured by western blot followed by densitometry using antibody against NQO1 (Santa Cruz biotechnology, Inc., California, USA) as described elsewhere [21].

### Cytochemistry

After surgically opening the femurs, bone marrow was aspirated by suction and expelled in small fractions on a number of microscopic slides and smears prepared. After air drying the smears were stained separately with Wright-Giemsa (Sigma-Aldrich, USA), Myeloperoxidase, Sudan Black, and Perls' stain (Merck, India) by standard procedures [68] and then examined under bright field microscope (Dewinter) equipped with high resolution digital Digieye 330/210 camera and Dewinter Biozard 4.1 software.

The article "NAD(P)H: Quinone Oxidoreductase 1 Deficiency Conjoint with Marginal Vitamin C Deficiency Causes Cigarette Smoke Induced Myelodysplastic Syndromes" was retracted in 2026. Reasons: duplicated data; overlap with earlier publications; original data or images not available; unreliable results or conclusions.

### Histology of bone marrow

The bones were surgically removed, placed in 10% neutral buffered formalin for 24 hours, decalcified in 7.5% formic acid for 72 hours and then processed routinely [21]. The tissues were embedded in paraffin, subjected to microtomy at 5 µm and prepared routinely for hematoxylin and eosin (H&E, Merck, India) staining and analyzed under bright field microscope (Dewinter).

### Measurement of CD34+ cells

Bone marrow cells were aspirated in phosphate buffered saline (PBS), fixed in 2% paraformaldehyde, pH 7.4, followed by permeabilization. Then blocking was done with 5% BSA in PBS solution for 1 hour at room temperature. After two washes in PBS, primary antibody against CD34 (Santa Cruz biotechnology, Inc., USA) was added and incubated over night at 4°C. The cells were then washed and incubated with FITC conjugated anti mouse IgG for 1 hour and analyzed by FACS (FACS Caliber, Becton Dickinson, California, USA).

### Evaluation of chromosomal aberration

One hour after i.p injection of colcemid (0.04%, 10 ml/kg body weight), the bone marrow cells were aspirated in a hypotonic solution (0.075 M KCl) and evaluated for chromosomal aberration [21].

### Measurement of apoptosis

Apoptosis was measured by using the terminal deoxynucleotidyl transferase-mediated dUTP nick end labeling assay (TUNEL) [14] as well as by flow cytometry analysis (FACS) using Annexin V-propidium iodide (PI), as described previously [17].

### Immunoblot analyses

The bones of the experimental animals were cut, marrow flushed out, homogenized in lysis buffer containing 50 mM Tris-Cl (ph 7.4), 150 mM NaCl, 1 mM EDTA, 1 mM DTT, 1% NP-40, 0.5% Trion X-100, protease inhibitor cocktail (Sigma, USA) and phosphatase inhibitor cocktail 2 (Sigma, USA) [21] and then centrifuged at 19000 g for 15 minutes. Bone marrow lysates (75 µg protein) were separated on 10% SDS-PAGE, blotted on PVDF membrane, and probed with respective antibodies against p53, phospho-p53, Bax, Bcl-2, caspase 3, cleaved caspase 3, TNF-α, caspase 8, cleaved caspase 8, α-tubulin (Cell Signaling Technology, USA). For identification of p-BQ-protein adducts, lysates were prepared from bone marrow cells of MDS guinea pigs or bone marrow cells of sham control guinea pigs after incubation with aqueous extract of CS (AECS) for two hours *in vitro*, as described before [14], [17]. Then the lysates were immunoblotted using antibody (rabbit, polyclonal) against p-BQ. The antibody to p-BQ, raised in rabbit after immunization with p-BQ-bovine serum conjugant, was supplied by Abexome Biosciences, Bangalore, India.

### Measurement of ROS and oxidative damage

ROS was measured by flow cytometry (FACS Caliber, Becton Dickinson, USA) using dichlorodihydrofluorescein diacetate (H_2_DCFDA) as per manufacturer's (Sigma, USA) instruction. Data were acquired and analyzed using the CELLQuest Programme. Protein oxidation was measured by the formation of protein carbonyl using antibody to 2, 4-dinitropheny-hydrazine (DNPH) as per Oxyblot™ protein oxidation detection kit (Intergen, NY) described previously [14]. 8-oxodG was detected by immunofluorescence using antibody to 8-oxodG as per manufacturer's (Abcam, UK) instruction.

The article "NAD(P)H: Quinone Oxidoreductase 1 Deficiency Conjoint with Marginal Vitamin C Deficiency Causes Cigarette Smoke Induced Myelodysplastic Syndromes" was retracted in 2026. Reasons: duplicated data; overlap with earlier publications; original data or images not available; unreliable results or conclusions.

### Statistical analyses

All values are expressed as mean ± SD. Statistical significance was carried out using a two factor ANOVA, with factors being CS and DC/vitamin C, or one way ANOVA as needed. The p- values were calculated using appropriate F-tests. Difference with p-values<0.05 were considered significant.

## Supporting Information

Figure S1 **NQO1 expression in the bone marrow cells, indicating that there is no significant change in NQO1 expression at the protein level.** (Panel A) and (Panel B) Bone marrow lysates were separated by 10% SDS PAGE and subjected to immmunobloting using antibody against NQO1. Vit C means vitamin C.
(TIF)

Figure S2 **Differential staining of bone marrow cells showing myeloid hyperplasia and hypercellularity in MDS guinea pigs.** (Panel A) Bone marrow aspirates showing myeloid hyperplasia; magnification 200×. (Panel B) Bone marrow histology showing hypercellularity; magnification 400×. Vit C means vitamin C.
(TIF)

Figure S3 **Signal transduction and cell cycle analyses in MDS guinea pig at different periods.** (Panel A) EGFR was immunoprecipitated (IP) with anti-EGFR and the precipitated proteins were immunoblotted (IB) with anti-phospho-Try (PY20) and anti-EGFR. (Panel B) Immunoblots of HRAS+KRAS, ERK1/2, p-ERK1/2, c-Myc, p-c-Myc, Akt and p-Akt.; p-EGFR, phospho-EGFR; p-ERK1/2, phospho-ERK1/2; p-c-Myc, phospho- c-Myc; p-Akt, phospho-Akt. (Panel C) Cell cycle analyses of bone marrow by flow cytometry: Y-axis, cell counts; X-axis PI stain. M1 represents G0/1; M2, S; M3, G2/M- phase. Vit C means vitamin C.
(TIF)

Table S1 Peripheral blood cell count of different treated male guinea pigs.
(DOC)

Table S2 Myeloid and Nonmyeloid cell ratio in bone marrow.
(DOC)
